# Unleashing the role of e-word of mouth on purchase intention in select Facebook fan pages of smart phone users

**DOI:** 10.1371/journal.pone.0305631

**Published:** 2024-09-03

**Authors:** Mohammed Arshad Khan, Syed Mohd Minhaj, Vivek, Mohammed Alhashem, Mohammed Kamallun Nabi, Mohd. Afzal Saifi, Asra Inkesar

**Affiliations:** 1 Accounting Department, College of Administrative and Financial Sciences, Saudi Electronic University, Riyadh, Saudi Arabia; 2 Department of Commerce, Jamia Millia Islamia, New Delhi, India; 3 Department of management, College of Administrative and Financial Sciences, Saudi Electronic University, Riyadh, Saudi Arabia; 4 Centre for Distance and Online Education, Jamia Millia Islamia, New Delhi, India; Al-Ahliyya Amman University, JORDAN

## Abstract

**Objective:**

This study aims to examine the impact of e-WOM on customer purchase intentions in Facebook fan pages using theories of trust, value co-creation and brand attitude. The present research has set out to explore this emerging domain of study and has thus developed & tested propositions which attempt to establish a relationship between e-WOM and customer‘s purchase intentions. A deeper understanding of this possible association is obtained by studying the mediating roles of Trust, Value Co-Creation, Brand Image and Brand Attitude.

**Methodology:**

The context for exploring this phenomenon is chosen to be the fan pages of smartphone brands on Facebook. The study involved conducting a sample survey of 490 respondents, comprising of both male and female, who belong to 5 smartphone brands Facebook fan pages–Samsung, Moto G, Lenovo, MI and ASUS are considered for the study. Out of which sample of 100 each has been targeted individually

**Findings:**

The findings suggested that e-WOM significantly predicts the purchase intentions of the customers of a specific product and considerable impacted on the purchase decision. The findings of the study also reveal that customer ‘s trust beliefs, perceived value co-creation, brand image and brand attitude partially mediate in between relationships of e-WOM and purchase intention

**Conclusion:**

The actual presence of different types of consumer electronics brands on the social media, more prominently, the smartphones, which undoubtedly are the most ubiquitous product of this segment. In fact, this indicates that presence on social media is a well- thought organizational strategy developed by companies to gain partial control over the customer ‘s decision- making process by establishing a close connect with the customers for a long period.

**Implication:**

This consequence will significantly impact the decision-making process of marketers or practitioners in relation to their marketing tactics. This research also indicates that marketers could devise more effective methods for distributing marketing content through social networking sites, while corporations can cultivate favorable electronic word-of-mouth for their products or services. Through the implementation of social media marketing strategies, companies can increase their sales volume and generate higher revenue. The study examined the role of trust, virtual community participation, and desire to purchase as mediators on smartphone brand fan sites on Facebook. It was observed that these factors had a partial influence on customer purchase intention.

## 1. Introduction

Over the past decade, social media has experienced tremendous growth, and this vast expansion has enabled it to operate in the realm of business as a critical promotional instrument that has the potential to connect to the customers at a personal level. Organizations have changed their marketing strategies and chosen the interactive platform of social media over the traditional marketing practices [1]. Through abolishing the need for a middleman in online transactions, social media has become an integral part of the decision-making process by giving constant, relevant peer input at every stage of the buying process.

Social networking sites (SNSs) have tremendously affected the way organizations perform business as well as the social and virtual lives of the general public [2]. Social networking sites enable users to make their own websites where they may share and discuss their own experiences in both the online and offline worlds. SNSs give an opportunity to the customers to communicate and exchange information and knowledge to create and keep up social connections; and to build up interpersonal, organizational ties [3]. Similarly, Social networking sites permit businesses to spread market information and engage customers by means of brand/fan pages. Organizations have leveraged the potential of fan page platforms to build strong associations with their customers. From a managerial point of view, fan pages may facilitate better management of customer relationships. The online brand fan pages are an open door for the organizations to discover what their customers think about the brand. Virtual fan pages have a significant influence on consumer behaviour as the feelings and opinions of other shoppers are conspicuous during purchases [4].

Other social networking sites like Twitter, Instagram and LinkedIn have a significantly smaller user base in comparison. Promoting a product’s reputation in the minds of consumers can be costly, but social media brand platforms provide a low-cost alternative. Therefore, in the recent past, a few studies have been directed to explore how eWOM is developed and how it influences consumer behaviour in social networking media [5]. Web-based social media might be categorized into various classe [6]. In light of the existing media speculations, [7] classified web-based social media into six classes:

1. Social network sites (SNSs), i.e., Facebook and Twitter etc.
2. Virtual content-sharing communities, i.e., YouTube and Wikipedia etc.
3. Blogs,
4. Electronic forums,
5. Virtual games world,
6. Content aggregators.

[8] have come up with honeycomb model, which portrays ―seven useful building pieces of social media ―discussions, sharing, identity, presence, connections, fame and gatherings‖. Each one of these building blocks presents functional utility for the user, which is derived from the various types of social media. For example, Facebook is a virtual communication networking site, and its core functional utility is "social relationships", "reputation building" and "conversations". Marketers derive utility from social media based on its classification. Social media involves the use of various tools such as online chat rooms, YouTube, Facebook, blogs, Twitter, Facebook, LinkedIn, Google etc. Utility inferred by marketers might be enhanced customer service, brand engagement and electronic word-of- mouth referrals [5].

### Problem statement

The social nature of social media is unique and is an interesting setting for investigating consumer behaviour. Consumers present in online platforms generate a tremendous amount of e-WOM through product reviews, opinions, feedbacks and recommendations, thus influencing consumers in their social networks as well as other consumers by stimulating a specific type of perception towards that product and thus redirecting their purchase-decisions.

In addition, studies have majorly focused on antecedents of online product-related experience sharing and less on the outcomes, thus providing scope for additional research. Also, only limited theories have been utilized to explain consumer behaviors in social media. For e.g., trust theory and value co-creation theories have previously been applied to study the influence of e-WOM on intentions to purchase.

**A significant contribution** can be made by viewing the concept of e-WOM under the lens of other theoretical perspectives. More specifically, while studying the most ubiquitous social network with the presence of multiple brands, i.e. Facebook, theories from social psychology such as social capital theory have been used as a foundation, indicating the potential of theories from social psychology to explain phenomena related to e-WOM. It was also observed that most studies ignored the impact of e-WOM in shaping the brand image of a product which is a significant gap given that brand image communicates the product quality.

### Research purpose

This study aims to examine the impact of e-WOM on customer purchase intentions in Facebook fan pages using theories of trust, value co-creation and brand attitude. To examine how these components inter-relate with each other and these relationships are supported by relevant literature review. The proposed framework indicates that e-WOM has direct and indirect effects on consumer purchase intentions, and it is mediated by value co-creation, trust, brand attitude and favorable hedonic and functional brand image of underlying products. With increasing significance of the present trends in the virtual brand communities ‘literature and the ceaseless relevance of web-based social networking environment for marketing practice, this research especially centers around the brand fan pages embedded in Facebook relationships between e-WOM and purchase intentions.

### Motivation and novelty of the study

Social media serves as a means to engage with customers in the contemporary marketplace and holds significant untapped potential for organizations. Due to its importance for businesses, scholars view it as a research area that can help them analyze practical issues and offer practical solutions.

This has resulted in a deeper comprehension of two aspects: the impact of peer influence on customer decision-making on social networking sites (SNSs) and the potential for generating greater value. The study provided valuable insights into the significance of customer involvement on online platforms, specifically within the context of Facebook users. This study not only adds to the existing body of research on electronic word-of-mouth (eWOM), but also advances the understanding of value co-creation by examining its relationship with eWOM and purchase intention, which has not been previously investigated. The findings also indicate that marketers should align themselves with consumer advocacy and strive to offer pertinent and all-encompassing information to customers in order to foster positive electronic word-of-mouth (eWOM), which will cultivate a favorable perception of their companies.

### Rationale for the study

Unique in its social nature, social media provides an intriguing environment in which to examine consumer behavior. The burgeoning popularity of social networking sites (SNSs) is fundamentally altering the way in which products endure in the marketplace. Consumers who are active on online platforms contribute a substantial volume of electronic word-of-mouth (eWOM) via product evaluations, recommendations, opinions, and feedback. This eWOM has the ability to sway consumers within their social circles and other consumers by inducing a particular type of perception regarding the product in question, thereby altering their purchasing choices.

It was also noted that the majority of studies disregarded the influence of eWOM on a product’s brand image, a significant omission considering that brand image conveys information about the quality of the product. An escalating number of consumers are consulting online sources of information prior to making purchases. This is particularly apparent with regard to intricate products such as smartphones. Given this situation, the majority of smartphone manufacturers have established fan profiles on social networking sites to ensure their presence. SNSs, such as Facebook, have evolved into a venue for consumers of all types, whose purchasing habits and requirements vary.

### Structure of the paper

Section 1: This section gives a brief introduction to the study and provides a Problem Statement, significance, and Research Purpose of the study.
Section 2: This section presents a literature review related to eWOM, VCC, Trust beliefs, Brand attitude and Purchase intentions in the context of smartphone brands present in SNSs in India. It is also covering the research gaps, research questions, and objectives of the study.
Section 3: This section presents a hypothesis development of the study.
Section 4: This section deals with the research methodology adopted in the study. It covers

research design, sampling, questionnaire design and data collection, data processing, data

analysis using statistical techniques.

Section 5: This section explains the data analysis’s and results of Exploratory Factor Analysis (EFA) and Structural Equation Modeling (SEM).
Section 6: This section presents the conclusion of the study. After consolidating the approach followed and results derived in the research study, it offers the discussions of the findings along with theoretical and managerial implications. It finally concludes

## 2. Literature review

Previous studies have shown that user-generated electronic word-of-mouth created by the customers, significantly influences consumer behaviour. In particular, the research on e-WOM offers various perspectives on the influence of e-WOM on consumer behaviour. The group of researchers identified a unique impact of e-WOM on customers behaviour (e.g., Customer value, loyality, purchase intention etc. [9].

Similarly, e-WOM on social media is shown to influence consumer attitude towards products. Earlier studies have demonstrated that customers are more likely to follow the recommendations of their peers than those of merchants [10]. Moreover, studies identified that e-WOM has a major impact on consumer opinion on the product judgment, loyalty and purchase behaviour [11]. Specifically, under e-WOM concept "content and source of e-WOM" has been studied widely. Notably, studies have shown that both positive and negative and there is a substantial effect of e-WOM on consumer behavior. In particular, both positive and negative e-WOM have a significant impact on consumers’ propensity to make a purchase [12].

[12], noted that co-creation is the process, where firm and customer jointly co-create value and specifically various factors are majorly contributed by the consumers in the process of co-creating value [13] identified that customer-to-customer interactions determine value co-creation in the virtual community and have positive effects on C2B, C2C relationships as well as on purchase intention and brand loyalty. [14] also elaborated the value co-creation theory and the concept of virtual engagement platforms to analyze the customer purchase behaviour and to contextualize the co-creation experiences [15].

Overall, the survey research found that the consumer comments generated on Facebook show a Significant impact on the decision-making process of customers [16], identifies the effect of social network media users comments on possible consumers purchase intention. The research surveys used the major SNSs platforms, for example- Facebook, Instagram, and Youtube [17]. The study combined the two theories of Information Adaption Model (IAM) and Theory of Reasoned Action (TRA) to understand consumer purchase intention. SEM results found that social integration has a significant influence on consumers purchase intention through perceived trust and brand attitude [18].

A consumer who receives information from the peers relating to product or services can be influenced by their opinion and has a high probability of greater purchase intention as the consumer believes the source credibility [19]. In this way, word- of-mouth is viewed as a critical tool to provide information and to reduce ambiguity before the purchase of products or services. The purchase intentions towards products or services are a subject of WOM [20]. If the source gives positive information about the products (i.e. positive WOM), consumer purchase intention become very high. If the source provides negative information about the products, during that time consumer purchase intention tend to be low [13].

In the value co-creation process, both the supplier and the client contribute to the value of the final product or service through their unique sets of skills and knowledge [21] conceptualized this notion as the shared trade of learning among the consumer and seller. According to their definition, value co-creation is the process through which a company’s customers and its employees work together to improve an existing product or service. [21], also assume that when a customer engages emotionally with a brand, such engagement of the consumer leads to value co-creation [22]. It is claimed that e-WOM influences consumers’ intent to buy products in two ways: directly and indirectly through users’ value co-creation activities. As we’ve seen, informal electronic communication from customers is just another way that people interact with social networking sites. Value co-creation in this process is profoundly affected by customer-generated e-WOM [23].

In addition to that, a recent study explains the VCC experiences generated through C2C interactions among online community members [24]. The review has proposed an interactional model of C2C activities between community members to engage in VCC collaboratively [25]. Similarly, [16] SNSs fan pages are the platforms for VCC activities where ― There is no point in maintaining an SNS fans page if no one is going to see it or use it. Customers’ actions, such as visiting the SNS fans page to learn more about the product and leave feedback, contribute to the page’s value [26].

### 2.1 Research gap

Initially, it is clear from the review of previous studies that only limited attempts were made to associating Facebook fan pages with e-WOM. Some prior thoughtful review investigations have found a connection between e-WOM and SNSs [27], mostly focused on the use of e-Forums, blogs, chatbots etc. and as a platform for e-WOM analysis [28]. Few researchers have mainly studied e-WOM engagement behaviour as comprised of online as well as offline activities [29]. They tend to consider social networks alone and are not focused on social networks devoted to specific brands. According to the trust theory and the “technology acceptance model (TAM)”, studies on the idea of e-WOM noticed that influences consumers’ trust and, in turn, their desire to make a purchase. Moreover, it also identified that e-WOM affects value co-creation and trust on the product, which further changes purchase intention. This is seen as proof that value co-creation acts as a mediator between e-WOM and intent to buy. There is evidence that e-WOM has a favorable effect on consumer intent to buy as a result of changes in brand attitude and brand image Brand image is categorized as hedonic and functional brand images which will also affect purchase intention in SNSs [30].

### Research questions

RQ 1: How does e-WOM affect consumer purchase intentions in Facebook fan pages of smartphone brands?
RQ 2: Does trust belief on product/brand affect the purchase intentions?
RQ 3: How does trust belief formed by e-WOM affect value co-creation and how such value co-creation ultimately affects purchase intentions?
RQ 4: Whether hedonic or functional brand image has any impact on direct relationship between eWOM and purchase intentions?
RQ 5: What role does brand attitude play on the direct relationship between eWOM and purchase intentions?

### Objectives of the study

1. To examine the effect of eWOM on consumer purchase intentions in Facebook fan pages.
2. To examine the effect of trust belief that is formed by eWOM on consumer purchase intentions.
3. To find out the effect of hedonic and functional brand image formed by eWOM on consumer purchase intentions.
4. To examine the effect of brand attitude formed by eWOM on consumer purchase intentions.
5. To explore the simple mediation effect of trust belief, value co-creation, brand attitude and hedonic & functional brand image on the direct relationships between eWOM and purchase intentions.
6. To explore the serial mediation effect of trust belief, value co-creation on the direct relationships between eWOM and purchase intentions.

## 3. Hypothesis’s development

### 1. The Relationship between e-WOM and purchase intention

Existing scholarly research has argued that e-WOM via online networking has an effect on consumers’ propensity to make a purchase. According to studies conducted by [31], consumers frequently rely on online evaluations or queries before making a purchase decision. To be more specific, word-of-mouth (e-WOM) in online marketplaces can affect the cost of both costly and economical goods and services [32]. The same is true on “Facebook fan pages”, where user-generated information like “comments, likes, shares, and feedback” has a significant impact on consumers’ propensity to make a purchase. Thus, this study derives the following hypothesis:

H1: e-WOM in Facebook fan pages has a positive effect on consumers purchase intention.

### 2. The Relationship among the e-WOM, trust, value co-creation and purchase intention

The context of their conceptual paper, [33] define co-creation as a value-creating process that includes the customer, the supplier, and the firm. They also state that open customer engagement with a brand helps the customer acquire more about the product or service and ultimately leads to a higher likelihood of purchase. In light of this, VCC now includes spoken electronic communication as a form of client engagement on SNSs. This procedure is strongly influenced by e-WOM generated by customers, which in turn affects esteem co-creation. According to [34], the first step in VCC is for a company to establish an interactive platform in the form of a social networking service (SNS) fan page in order to cultivate the brand image and disclose market information. For businesses, customer actions will lead to better two-way communication and new chances to expand and enhance existing offerings. Fan pages increase VCC by virtue of the e-WOM interactions with customers; positive e-WOM boosts company credibility and gets more people involved with brands [35].

As stated, e-WOM is a variable influencing buyers’ trust in the firm and its goods and services. We expect that e-WOM directly affects value co-creation through trust on products in Facebook fans pages. Furthermore, value co-creation effects purchase intention [36]. Here, conviction in the firm (or trust) is the determining factor in the co-creation of esteem. Turning to trust in integrity, positive e-WOM in fan pages strengthens the trust in integrity when a firm provides quality goods and services as it promised, whereas negative e-WOM reduces such beliefs. Thus, the study derives the following hypothesis.

H2: e-WOM in Facebook fans pages has a positive effect on consumer trust belief on brand.
H3: The level of consumer trust belief on brand will have positive affect on Value co- creation in Facebook fan pages.
H4: e-WOM in Facebook fans pages has a positive effect on Value co-creation.
H5: Value co-creation has a positive effect on consumer purchase intention.

### The relationship of trust belief with brand attitude and purchase intention

In turn, the trust concept has been studied by relating with brand attitude in the past, particularly in the online setting [37]. Online environment reviews play a significant role in consumer purchase decision. These numerous reviews help and reduce uncertainty during consumer buying decisions process [38]. Among the innumerable studies, consumer-generated reviews are more credible than firms [39]. On the other hand, e-WOM source credibility may reduce trust in sellers if the consumer perceives that the seller’s website consists of incomplete or biased information, which leads to negative trust towards the seller.

[10], state that trust in sellers significantly influences consumer purchase intention from the same e-commerce website again. [40] noted that trust in online sellers directly affect consumer attitude towards the product because consumers perceive that the product has more benefits and can avoid possible risks from the online purchase. We expect that with the influence of online reviews in social media fan pages, consumers trust increases on brands and such brand trust affects consumer purchase intention.

H6: The level of consumer Trust belief on brand will have positive affect on consumer purchase intention in Facebook fan pages.
H7: The level of consumer Trust belief on brand will have positive affect on brand attitude in Facebook fan pages.

### The relationship between e-WOM and brand attitude

Studying the effect of e-WOM via social media can also be done by gauging consumers’ feelings and intentions toward a brand. Marketers have long recognized the power of word of mouth in shaping consumer opinion of a product or service and their propensity to buy it [41]. Similarly, the firm hosted fan pages consumers generated positive comments heighten the favarable attitude towards the brands, in contrast to that negative comments lead to a hostile attitude towards the brand. Purchase intention interpreted as an individual’s likelihood of buying a specific product. Thus, the following hypothesis is as follows:

H8: e-WOM has a positive effect on brand attitude in Facebook fan pages
H9: Brand attitude has a positive effect on purchase intention in Facebook fan pages

### The influence of e-WOM on hedonic and functional brand image

As specified before, the present study investigation takes as a base attribution theory to comprehend the impacts of e-WOM in SNSs on customer brand image. Brand image is one of the marketing strategies to differentiate the brand from the competitive brands. Someone’s perception of a brand can be defined as their "beliefs, ideas, and impressions" of that brand [42]. Online reviews, user comments, likes and sharing, text on blogs and user usage experiences more effective in creating a brand image than oral communication. According to [43], consumers can evaluate a brand’s reputation by gauging how positively they feel about the product’s features and benefits. Two subcategories of brand identity, "functional" and "hedonic," have been identified. Brand performance and its utility are measured through the Functional brand image.

Whereas, hedonic brand image stresses the customer feelings and emotions associated with the brand. Perceived usefulness of online reviews also influences the functional brand image. Therefore, it is noted that Facebook fan pages generated user content in the form of likes, sharing, comments and posts creates the functional and hedonic brand images towards the products that are offered for sale on the market and which will turn into consumer purchase intention. Thus, hypothesis is articulated as:

H10: e-WOM has a positive effect on the Hedonic brand image in Facebook fan pages.
H11: Hedonic brand image has a positive effect on purchase intention.
H12: e-WOM has a positive effect on the Functional brand image in Facebook fan pages.
H13: Functional brand image has a positive effect on n purchase intention.
H14: Hedonic brand image is positively mediate on the direct relationships of e-WOM and consumer purchase intention.
H15: Functional brand image is positively mediate on the direct relationships of e-WOM and consumer purchase intention.
H16: The relationship between e-WOM and consumer purchase intention is mediated by brand attitude.
H17: The relationship between e-WOM and consumer purchase intention is mediated by the trust belief on brand.
H18: The relationship between e-WOM and consumer purchase intention is mediated by value co-creation.
H19: The relationship between e-WOM and consumer purchase intention is sequentially mediated by trust belief and value co-creation.

## 4. Research methodology

### Sampling strategies

The present study follows the cross-sectional design and a quantitative approach as the current research aims to measure the relationships between the hypothesized constructs in the proposed model in the backdrop of Smartphone brands in the social media context.

### Sample collection

Primary data was collected from members of the five smartphone fan pages via a self-administered online survey questionnaire.

The main study target population is members of the official fan pages of selected smartphone brands on Facebook. Specifically, the sample constitutes both male and female respondents who belong to the five fan page groups under single product category. There are a couple of difficulties associated with the selection of the population. As indicated by a few sources, Facebook has around 1.95 billion dynamic Facebook users in 2021 [44]. Fan page followers grow continuously; there is no definite population in the fan pages. Due to the existing limitations, the study decided to use a purposive sampling technique to collect the data.

There are no particular rules when determining sample size for non-probability sampling; instead, it regularly relies upon various specially appointed methodologies, including general guidelines proposed by different researchers, in addition to the budgetary constraints [45]. The sample size for the present study is determined based on the adopted methodology of analysis that is structural equation modelling (SEM).

### Measurement scaling

Initially, based on exploratory research, 11 fan pages of smartphone brands were identified, but based on the user base, number of comments and number of followers, this study identified the five leading and most active fan pages. The target population of the study were members of the five Smartphone brands fan pages on Facebook, who joined them and have been using them for the past one year. The study has selected five leading “fan pages of smartphone brands” (Samsung, Motorola, Asus, Apple and MI) in India. They were chosen based on the number of fans and the number of postings, “likes and comments” by the members. The success of fan pages can be assessed by a large number of fans, postings and number of posting by the fan members.

### Estimation techniques

The study uses three approaches–“exploratory factor analysis (EFA), confirmatory factor analysis (CFA) and structural equation modelling (SEM)”. Ruscio & Roche, (2012) suggests that when the proposed model is having less prior knowledge about theoretical model development; it is recommended to conduct EFA and CFA. Though the present research model does not have previous knowledge of structural development, it is assumed to conduct EFA before going to CFA. Accordingly, the study performs EFA to check the underlying structure of the conceptual model. Later CFA is performed to examine the “reliability and validity” of the model and also evaluate the goodness of fit indices of the research model.

## 5. Data analysis’s and results

The chapter, foremost, reports the demographic profile of the respondents who participated in this study, followed by descriptive statistics for each item on the measurement scale. Further, the chapter presents the outputs of “exploratory factor analysis (EFA), confirmatory factor analysis (CFA) and structural equation modelling (SEM)” in an elaborative manner.

Out of 490 respondents, 77.15% (378) of the respondents were male, and 22.85% (112) of the respondents were female as shown in Table 1.

**Table 1:** Demographic profile of the respondents.

Demographic Statistics			
Measure	Items	Frequency	Percentage
Gender	Male	378	77.15
	Female	112	22.85
Age	Up to 20	132	26.93
	20–30	108	22.04
	30–40	98	20
	40–50	85	17.34
	Above 50	67	13.67
Qualification	Intermediate	78	15.91
	Graduate	187	38.16
	Post graduate	115	23.46
	Professional degree	110	22.44
Internet access through most	Desktop/PC	95	19.38
	Laptop	105	21.42
	Smartphone	212	43.26
	Tablet	78	15.91
No of hours spend on internet per Week:	Up to 10 hours	201	41.02
	10–20 hours	97	19.79
	20–30 hours	103	21.02
	More than 30	89	18.16
News feeds received from Facebook fan page	Yes	410	83.67
	No	80	16.33
Post or comment on Facebook fan Page	Yes	381	77.75
	No	109	22.25

Table 1 represents the age of the respondents. 22.04% (108) of respondents were aged between 20–30 years, and almost 20% (98) of respondents were aged between 30–40 years, and 17.34% (85) of the respondents were aged between 40–50 and 26.93% (132) of the respondents were aged below 20 years and lastly 13.67% (67) of the respondents were aged 50 years above. Most of the respondents who participated in the survey belonged to the age group up to 20 years.

Table 1 represents the educational background of the respondents: Intermediate (15.91%), graduates (38.16%), postgraduate (23.46%), and Professional degree (22.44%).

Table 1 represents the Internet access available to the respondents through various devices: Desktop PC (19.38%), Laptop (21.42%), Smartphone (43.26%), and Tablet (15.91%). Among the respondents, the majority of the respondents– 43.26% were accessing the internet through Smartphone, and the least– 15.91% of the respondents were accessing the internet through the tablet.

Table 1 represents the amount of time spent on internet, Up to 10 hours (41.02%), 10–20 hours in a week (19.79%), 20–30 hours in a week (21.02%) and More than 30 in a week (18.16).

### 5.1 Data adequacy for factor analysis

Both the sphericity test by Bartlett and the sampling adequacy test by Kaiser-Meyer-Olkin (KMO) were confirmed, whether the research data variables are factorized efficiently. The observed co-relation matrix is compared to the identity matrix in “Bartlett’s test of sphericity”. It indicates a really significant disparity between the “observed correlation matrix” and the identity matrix [46].

The sampling adequacy (KMO) test compares the values of correlations that are partially correlated with each other. The result reveals that KMO is 0.861 (Table 2) and it is more than the “cut off value of 0.50” [47]. Thus, the adequacy test suggests that correlations between underlying constructs are sufficient to move for further analysis.

**Table 2:** KMO and Bartlett’s test.

KMO Sampling Adequacy		0.861
**Bartlett’s Test of Sphericity**	Approx. Chi-Square	76656.1
	Df	404
	Sig	0.00

### 5.2 Confirmatory Factor Analysis (CFA)

CFA is a part of SEM, which is applied to examine the measurement model and path estimates of the “structural model”. The present study CFA model is shown in Fig 1. The measurement model helps to define relationships of observed and unobserved variables. It identifies the pattern of each measurement factor loadings. CFA is conducted to validate the research model, and it is not meant for explaining the construct relationships. It explains how a measurement model variable is grouped to explain the particular constructs and applied to verify the reliability and validity. Therefore, the current study first checks the construct reliability and validity, and after that, the model fit indices were examined.

**Fig 1:** CFA model.

### 5.3 Construct reliability and validity

Construct reliability measures the internal consistency of observed, indicative variables. It clarifies whether all the variables measures are consistent on behalf of something. Construct reliability explains about the items or indicators of a construct. A construct is measured by its items or indicators as the theory defines. It is verified by “convergent and discriminant validity”. The convergent validity is calculated to find the convergence or correspondence among the similar constructs, while discriminant validity finds the discrimination among the dissimilar constructs.

#### 5.3.1 Construct reliability

“Construct reliability (C.R) is computed from the sum of the squared factor loadings of every construct and summation of error variance terms”. According to the Bentler & Bonett [48], to confirm the reliability of the factors, the C.R value of all the constructs should be above the cut off value of 0.7 is shown in the Table 3.

**Table 3:** Reliability of the constructs.

Constructs	Reliability
e-WOM	0.813
Purchase intention	0.863
Brand attitude	0.893
Value co-creation	0.818
Trust beliefs	0.930
Hedonic brand image	0.806
Functional brand image	0.762

#### 5.3.2 Convergent validity

“The extent to which two measures of the same concept are correlated" [49] is the definition of convergent validity (C.V). Standard loadings and the “average variance explained (AVE)” were identified by [50] as measures of convergent validity. [46] state that AVE > 0.5, CR > AVE, and CR > 0.70 are all necessary conditions for convergent validity.

#### 5.3.3 Discriminant validity

It’s the disparity between the similarities between two ideas and how different they actually are. Using AVE and MSV, we may evaluate the reliability of the factors [51] state the following conditions must be met in order to prove validity: “MSV < AVE and ASV < AVE”. The current study made sure that each construct ‘s “MSV and ASV were lesser than the AVE estimates”, which are shown in Tables 4 and 5.

**Table 4:** Construct validity and reliability.

Constructs	Cranach‟s Alpha	C.R	AVE	MSV	ASV
eWOM	0.813	0.822	0.541	0.289	0.135
TB	0.930	0.930	0.691	0.120	0.08
BA	0.818	0.818	0.600	0.094	0.056
PI	0.863	0.832	0.563	0.203	0.143
VCC	0.893	0.833	0.629	0.289	0.186
HBI	0.806	0.807	0.583	0.171	0.109
FBI	0.762	0.762	0.518	0.059	0.039

**Note: “**Construct reliability (C.R) > 0.70; Convergent validity (AVE > 0.5); C.R > AVE; Discriminant validity (MSV & ASV AVE); Square root of AVE > 0.70. Inter-construct relationship”.

**Note:** TB = Trust Belief, BA = Brand Attitude, PI = Purchase Intention, VCC = Value Co-

Creation, FBI = Functional Brand Image, HBI = Hedonic Brand Image.

**Table 5:** Discriminant validity.

Constructs	Ewom	TB	HBI	BA	PI	VCC	FBI
eWOM	**0.74**						
TB	0.254	**0.83**					
FBI	0.76	0.273**	**0.72**				
BA	0.76	0.302	0.402	**0.77**			
PI	0.76	0.093	0.193	0.179	**0.75**		
VCC	0.76	0.174	0.319	0.263	0.137	**0.79**	
HBI	0.76	0.209	0.356	0.343	0.170	0.188	**0.76**

### 5.4 Goodness of model fit

The most imperative part of CFA is to test the model of “goodness of fit indices”. Goodness of fit during model execution can be checked using maximal likelihood estimation (MLE) [52]. It is conducted to determine whether or not the model has a decent fit. There are various indices for evaluating model fit, such as chi-square divided by degrees of freedom (2/df), comparative fit indices (CFI), “Normed fit indices (NFI), Tucker-Lewis index (TLI), Root mean square error approximation (RMSEA), and root mean square residual (RMR)”.

The model was assessed by the following criteria: χ2/df< 3 GFI >0.8 [53]. As recommended by [51] (1980), “NFI > 0.90 and CFI ≥ 0.95, P should be near to 1 and RMSEA should be less than 0.5” [54] All the “model fit indices” fall under the accepted ranges with χ2/df = 1.826, “CFI” = 0.962, “GFI” = 0.917, “NFI” = 0.919, “TLI” = 0.956 and “RMSEA” = 0.041. Consequently, the values suggest that the “measurement model” is considered to be appropriate (Fig 2). Table 6 displays the goodness-of-fit indices for the investigation.

**Fig 2:** Common method bias using CLF method.

**Table 6:** Model fit indices.

Structural Model	Fit Statistics	Recommended Cut Off Values
CMIN/DF	1.826	< 3
P-VALUE	0.000	≥ 0.05
GFI	0.917	≥ 0.90
CFI	0.962	≥ 0.95
TLI	0.956	≥ 0.95
AGFI	0.898	≥ 0.80
NFI	0.919	> 0.90
RMSEA	0.041	≤ 0.05
P Close	0.999	Close to 1

### 5.5 Common method bias

In the suggested model, all of the “latent (factors) and manifest (items) variables” are examined simultaneously using a single questionnaire. Thus, it is possible that “common method bias” exists in the data. Single factor analysis was conducted in “IBM SPSS Version 25”. All of the indicators were entered into an unrotated EFA to see which factor explained the most variation. Common technique bias is represented by the single-factor variance [46]. As can be seen in Table 7, the Eigenvalue of the variation attributable to a single factor is 27.514, which is less than 50% of the threshold value. This indicates that the data is not affected by common technique bias.

**Table 7:** Harman single factor test.

Total Variance Explained						
Component	Initial Eigenvalues			Extraction Sums of Squared Loadings		
	Total	% of Variance	Cumulative %	Total	% of Variance	Cumulative %
1	8.008	27.614	27.614	8.008	27.614	27.614
2	3.332	11.491	39.105			
3	2.170	7.483	46.588			
4	1.888	6.509	53.097			
5	1.826	6.297	59.394			
6	1.668	5.751	65.14			
7	1.486	5.125	70.270			
8	.700	2.415	72.685			
9	.637	2.197	74.883			
10	.589	2.030	76.912			
11	.586	2.021	78.934			

We used AMOS Version-25 to handle the common variance. In the SEM analysis, we included the CLF creator variable and “compared the regression weights of the CLF with those of the confirmatory model elements”. According to Table 8, there are no significant differences in relative importance between three components. The CLF technique of common method bias is displayed in Fig 2, demonstrating that the study sample does not suffer from any common method bias.

**Table 8:** Results of Common Latent Factor (CLF) method for common method bias analysis.

Construct		Variables	Regression Weights without CLF	Regression Weights with CLF	Difference
Trust Beliefs	<‐‐‐	TB1	.872	0.826	0.046
	<‐‐‐	TB2	0.934	0.89	0.044
	<‐‐‐	TB3	0.823	0.772	0.051
	<‐‐‐	TB4	0.904	0.856	0.048
	<‐‐‐	TB5	0.744	0.68	0.064
	<‐‐‐	TB6	0.684	0.622	0.06
Value Co- Creation	<‐‐‐	VCC1	0.823	0.786	0.03
	<‐‐‐	VCC2	0.747	0.689	0.058
	<‐‐‐	VCC3	0.756	0.712	0.044
	<‐‐‐	VCC4	0.801	0.747	0.054
	<‐‐‐	VCC5	0.835	0.792	0.043
Purchase Intention	<‐‐‐	PI1	.779	0.73	0.049
	<‐‐‐	PI2	0.818	0.781	0.037
	<‐‐‐	PI3	0.791	0.746	0.045
	<‐‐‐	PI4	0.635	0.573	0.062
	<‐‐‐	PI5	.713	0.647	0.066
E-wom	<‐‐‐	WOM1	0.78	0.744	0.036
	<‐‐‐	WOM2	0.756	0.72	0.03
	<‐‐‐	WOM3	0.56	0.523	0.037
	<‐‐‐	WOM4	0.819	0.778	0.04
Brand Attitude	<‐‐‐	BTT1	0.743	0.695	0.048
	<‐‐‐	BTT2	0.777	0.739	0.038
	<‐‐‐	BTT3	0.802	0.748	0.054
Hedonic Brand Image	<‐‐‐	HB1	0.762	0.713	0.049
	<‐‐‐	HB2	0.807	0.769	0.038
	<‐‐‐	HB3	0.719	0.661	0.058
Functional Brand Image	<‐‐‐	FB1	0.715	0.657	0.058
	<‐‐‐	FB2	0.665	0.628	0.037
	<‐‐‐	FB3	0.774	0.729	0.04

### 5.6 Structural Equation Modelling (SEM)

SEM was conducted to verify the significance level of path coefficients to test the research hypotheses. The main objective of this analysis is to test the theory. The proposed research model should have sound theoretical. SEM technique is based on a covariance matrix to confirm the research model. It emphasizes the overall fit of the hypothesized covariance model with the observed covariance matrix [46].

The present study applied SEM to examine the path relationships between multiple constructs present in the research model. In line with the path analysis using SEM, the study also examines the structural model fit. This two-part analysis of structural equation modelling could help the study to carve out, whether the hypothesis is supportive or not supportive.

Table 9 shows the results of hypothesis testing including standard coefficients and path coefficients and their significance. Based on the significance of the “standardized coefficients”, i.e. (β) values, we can find supported hypothesis in the study. The un- standardized estimates and item loadings of each construct are evaluated for their significance. It also affirmed that item loadings of constructs are highly significant at the level of 0.001 (0.1%) and their P values. “The hypothesized inter- construct structural relationships and path coefficients (β)” are given in Fig 3.

**Fig 3:** Testing of hypothesis using path analysis.

**Table 9:** Results of hypothesis testing.

Independent Variable	Dependent Variables	Hypothesis	Standard Estimates (β)	Standard Error	t- Statistic	P-Value	Results
eWOM	Purchase Intention	H1	0. 199	0.067	2.995	0.003	Significant
eWOM	Trust Beliefs	H2	0.321	0.054	6.404	***	Significant
Trust Beliefs	Value Co- Creation	H3	0.187	0.041	4.155	***	Significant
eWOM	Value Co- Creation	H4	0.502	0.053	9.441	***	Significant
Value Co- Creation	Purchase Intention	H5	0.159	0.059	2.769	0.006	Significant
Trust Beliefs	Purchase Intention	H6	0.093	0.043	1.999	0.04	Significant
Trust Beliefs	Brand Attitude	H7	0.109	0.048	2.080	0.038	Significant
eWOM	Brand Attitude	H8	0.297	0.058	5.192	***	Significant
Brand Attitude	Purchase Intention	H9	0.190	0.051	3.775	***	Significant
eWOM	Hedonic Brand Attitude	H10	0.347	0.0.056	6.320	***	Significant
Hedonic Brand Attitude	Purchase Intention	H11	0.214	0.050	4.200	***	Significant
eWOM	Functional Brand Image	H12	0.221	0.050	3.904	***	Significant
Functional Brand Image	Purchase Intention	H13	.090	0.056	1.834	0.067	Not Significant

The analysis identified that “consumer-generated eWOM of Facebook fan pages has a significant effect on consumer purchase intentions” (β = .199 t = 2.995, p < 0.003 and so the respective hypothesis is supported (H1). eWOM significantly influences VCC (β = 0.502, t = 9.441, p < 0.001) and so the respective hypothesis is supported (H4). “It also suggests that VCC significantly influences consumer purchase intentions, which is validated” at (β = 0.159, t = 2.769, p < 0.006), hypothesis (H5). The hypothesis (H2) related to eWOM and Trust beliefs is significant at p < 0.001 with the value of β = 0.321, t = 6.404, and also Trust beliefs has significant influence on purchase intention (β = 0.093, t = 1.999, p < 0.046) (H6). The path coefficient of eWOM and brand attitude is β = 0.297, t = 5.192, significant at p < 0.001 (H8).

The path from Brand attitude to purchase intentions has significant effect with a value of (β = 0.190, t = 3.775, p < 0.001) (H9). The path from trust beliefs to value co-creation (H3) has significant effect with value of (β = 0.187, t = 4.155, p< 0.001). Trust beliefs significantly influences brand attitude (β = 0.109, t = 2.080, p < 0.038), and so the respective hypothesis is supported (H7). eWOM and Hedonic brand image have significant, hence hypothesis is accepted at (β = 0.347, t = 6.320, p < 0.001), (H10). Hedonic brand image significantly influences purchase intention (β = 214, t = 4.200, p < 0.001) and so the respective hypothesis is supported (H11). eWOM significantly influences Functional brand image (β = 0.221, t = 3.904, (p < 0.001) and so the respective hypothesis is supported (H12). On the other hand, Functional brand image shows insignificant influence on purchase intention (β = 090, t = 1.834, p < 0.067, and so the respective hypothesis is not supported (H13). All the remaining hypotheses in the research model, except H13, were supported.

### Serial mediation effect of trust beliefs and value co-creation on eWOM and purchase intentions (H19)

In the present study, all the path parameters were estimated simultaneously in the structured path model and serial mediation. The study has examined three path mediation effects in Table 10. According to the Gruen, T. W., Osmonbekov [30], this approach facilitates researchers to detach both the indirect mediation effects of Trust beliefs and Value co-creation. This method also allowed us to investigate the linked effect via two of these mediators (H19). In order to evaluate the validity of the suggested model, the present study employed a process macro utilizing the SPSS version-25 software to conduct Tests of the "Three-Path Mediated Effect". According to the Vargo, S. L., Maglio [12], the analysis of Organizational Research Methods and mediation is conducted using a bootstrapping procedure, instead of test procedure because it is efficient than any other procedure for the testing of indirect effects.

**Table 10:** Mediation analysis results.

Independent Variable	Dependent Variable	Standard Total Effect	Standard Direct Effect	Standard Indirect Effect	Results
H14: Hedonic Mediator Effect on Brand Image (HBI)					
Ewom	HBI	0.403***	0.403***	0.0	Partial Mediation
HBI	PI	0.405**	0.405**	0.0	
eWOM	PI	0.510	0.510	0.092	
H15: Functional Mediator Effect on Brand Image (FBI)					
eWOM	FBI	0.205	0.205	0.0	Partial Mediation
FBI	PI	0.181	0.181	0.0	
eWOM	PI	0.511	0.511	0.031	
H16: Mediator Effect with respect of Brand Attitude (BA)					
eWOM	BA	0.307	0.307	0.0	Partial Mediation
BA	PI	0.259	0.259	0.0	
eWOM	PI	0.450	0.370	0.08	
H17: Mediator Effect with respect of Trust Belief (TB)					
eWOM	TB	0.231	0.299	0.0	Partial Mediation
TB	PI	0.189	0.191	0.0	
eWOM	PI	0.501	0.401	0.055	
H18: Mediator Effect with respect of Value Co-Creation (VCC)					
eWOM	VCC	0.449	0.498	0.000	Partial Mediation
VCC	PI	0.279	0.301	0.000	
eWOM	PI	0.501	0.311	0.153	

As predicted in H1, eWOM is positively related to purchase intentions. H17 assumed that the Trust beliefs mediate between “eWOM and Purchase intention”. This hypothesis was also found significant. H18 was supported that the VCC mediates the path from eWOM to Purchase intention. H19 mentioned that Trust beliefs and VCC sequentially mediated the direct path “relationship between eWOM and purchase intention”. The hypothesis revealed that eWOM in Facebook fan pages enhances the trust in products and also promotes VCC activities, which ultimately affects the consumer purchase intentions.

## 6. Discussion

### The relationship between eWOM and purchase intentions (H1)

Understanding the impact of electronic word of mouth (eWOM) on Indian smartphone manufacturers is the goal of this study. The influence of eWOM on Facebook fan page followers on purchase intention of Smartphone brands was found to be significant (H1). Consumers’ desire to buy a product was found to be significantly influenced by user-generated information on social media, such as likes, comments, shares, and so on, according to a research of smartphone companies. The hypothesized "relationship between eWOM and purchase intentions" is consistent with the earlier findings of etc. [55]. The authors indicated that the construct eWOM is the most influential element determining customer "purchase intention" in an online setting.

### The relationship of trust belief with eWOM, brand attitude and value co- creation (H2, H3. H5, H6, H7, H17, H19)

There was a statistically significant favorable effect of eWOM on brand trust perceptions (H2). The current study reveals that customers active participation in Facebook fan page community activities (such as like, comments, “posting and reviewing smartphone brands” information and brand experiences and actively engaging in fan page activities) were integrated with trust towards smartphone brands. The outcome agrees with those of [56] proposed the link between eWOM and trust belief and noted that consumer-generated content (e.g., positive comments, likes, posts) would form a positive trust belief on products/services of a brand and further leading to purchase intention.

In addition, the "direct relationship between eWOM and purchase intentions" is mediated in a favorable way, according to the study, by consumers’ levels of Trust confidence in a company (H17). This result is in line with the findings of [57] noted that the customer who highly engages (reading comments and posting) in eWOM on social media fan pages tend to develop trust towards the brands customers on fan pages support each other on the usage of products or services of a particular brand.

The positive effect of trust beliefs on VCC (H3) and VCC activities on purchase intention (H5) in smartphone brands in Facebook fan pages were found significant in the current study. These results specify that active customer engagement in eWOM activities enhances the trust in brands, which consequently lead to VCC and produce positive purchase intention.

The results for hypothesis H3, H5 are supportive of the notion of [58], who posited that the customer trust beliefs positively affect VCC and purchase intention. Facebook fan pages of smartphone brands also show a substantial (H6) connection between trust beliefs and intent to buy.

The results also support the notion that there is a positive link between trust beliefs and brand attitude (H7) is significant. It indicates that the active customer engagement in fan pages builds the trust in the brand, which leads to favourable or unfavourable intention towards the brand [59]. The study additionally examined how trust beliefs and VCC mediate the “The impact of eWOM on consumer behavior inside fan communities” (H19). It was discovered that consumer purchase intentions are significantly influenced by a favorable partial mediating effect.

### The relationship of value co-creation with eWOM and purchase intentions (H4, H5, H18)

The data corroborated the hypothesis (H1) that eWOM influences consumers’ intent to make a purchase (the route link between eWOM and intent to purchase was statistically significant). In addition, VCC (H4 and H5) is a major channel via which eWOM affects consumers’ propensity to buy. It follows that favorable eWOM spread via fan pages boosts VCC and consumer intent to make a purchase. Facebook fan pages for Smartphone manufacturers facilitate two-way communication with consumers through positive feedback and sharing. These connections aid businesses in developing new products and refining existing ones.

In this study, we found that VCC does, in fact, somewhat mediate the relationship (H18) between eWOM and intent to buy. Results from this study agree with those from prior research [60]. By putting the hypothesized eWOM SNSs to the test, these results also provide credibility to the existing theoretical frameworks.

### The relationship of brand attitude with eWOM and purchase intention (H4, H6, H8, H16)

The association between eWOM and Brand attitude (H8) from smartphone companies Facebook fan pages members were discovered significantly positive. Additional results from "the study show that the influence of brand attitude on purchase intentions was found to be significant" (H9). The present study investigates the favorable association between electronic word-of-mouth (eWOM) and brand attitude specifically within the context of smartphone fan pages (H6) is in line with the findings of [61]. This association indicates that sharing content on Facebook fan pages can significantly influence prospective buyers’ decisions to make a purchase.

Participants of Facebook fan pages had a generally positive view of brands. The relationship between eWOM and consumers’ intent to buy is mediated by their feelings about the brand (H16). Accordingly, the result of the current study found brand attitude as a significant factor that enhances the consumer engagement activities with brands and increases the purchase desire on “Facebook fan pages of smartphone brands”.

### The relationship of hedonic and functional brand image with eWOM and purchase intention (H10, H11, H12, H13, H14, H15)

Moreover, "the effects of eWOM on intentions" to purchase were examined via the lens of brand perception in this study. Brand reputation can be broken down into the First Impression (FBI) and the Halo Effect (HBI) [62]. The current research used a cross-sectional design to test for the predicted associations, and it reveals that eWOM has a considerable positive affect on the hedonic and functional brand images in Facebook fan pages (H10, H11). From revealed results, it seems that Facebook fan pages consumers are more influenced by the HBI on purchase intentions (H11). In contrast, the influence of FBI which is formed by eWOM on fan pages has an insignificant effect on purchase intentions (H12, H13). It denotes that the utility, efficiency and effectiveness of smartphone brands are not effective on “consumer purchase intention”. Further, the study conducted mediation effect of both kinds of brand images on the “influence of eWOM on purchase intentions” (H14, H15) and found significant mediation effect on the direct relationships among constructs in the social media fan pages. The results of this investigation are consistent with those of [31].

## 7. Theoretical and practical contribution

Social media serves as a means of connecting with clients in the contemporary economy and holds significant untapped potential for enterprises. Due to its importance for businesses, researchers believe it to be a field of study that allows them to analyze practical problems and offer practical answers (Kaplan & Haenlein, 2012). Therefore, the present study holds great importance from both a theoretical and practical standpoint. This study examines the impact of online reviews or electronic word-of-mouth (eWOM) on brand image and purchase intentions for a product by including the Theory of Reasoned Action (TRA), Theory of Planned Behavior (TPB), Technology Acceptance Model (TAM), and Attribution Theory. The proposed model is based on trust theory and value co-creation theory. It aims to examine the impact of a customer’s trust in a brand on their communication behavior on social media. Additionally, it explores how marketers and customers can collaborate to create more value by developing improved products through continuous feedback via electronic word-of-mouth (eWOM). This has resulted in a deeper comprehension of two aspects: the impact of peer influence on customer decision-making on social networking sites (SNSs) and the potential for generating greater value.

## 8. Managerial implications

The results will be useful in the improvement of marketing strategies by using social media fan pages to improve VCC process with their prospective customers. These findings can help practitioners to implement VCC in SNSs and to encourage customers to repeat intention to purchase of their products or services. By applying social media marketing practices, firms enhance sales volume and revenue. Trust, virtual community engagement, and intention to purchase were all investigated as mediators on smartphone brand fan pages on Facebook, and found a partial impact on the consumer purchase intention. Reviews, comments, and feedback from customers have been shown to significantly influence purchasing decisions. This outcome will have an influence on marketers or practitioners decision-making process regarding their marketing strategies. This research also suggests marketers develop better ways to disseminate marketing information through social networking sites and firms can develop positive e-wom for their products or services.

Managers may learn more about their customers and use social media to boost their company’s reputation by monitoring fan sites on Facebook. The study’s results can help them develop a novel strategy for spreading product information via SNSs. Considering favorable eWOM will in turn affect purchase decisions, this research can also be valuable for boosting public opinion of companies and services.

## 9. Conclusion

Social media has facilitated interactions between firms and their customers, enabling consumers to actively engage in the process of value co-creation (VCC). However, one must use the platform carefully as the consequences are shared. The literature indicates that organizations utilize social media to convey their products and brand messages. However, it is crucial for them to recognize the significance of customer feedback in the form of opinions, discussions, feedback, and arguments. This information has the potential to forecast the purchasing behaviors of other customers, provided that it is effectively managed.

The study’s core findings indicate that eWOM in well-known SNSs include as―Facebook, had a significant impact on dependent variables: value co-creation, trust beliefs, brand attitude, brand image and purchase intentions. This finding lends support to the actual presence of different types of consumer electronics brands on the social media, more prominently, the smartphones, which undoubtedly are the most ubiquitous product of this segment. In fact, this indicates that presence on social media is a well- thought organizational strategy developed by companies to gain partial control over the customer ‘s decision- making process by establishing a close connect with the customers for a long period.

Additionally, consumer behavior outcomes in relation to mobile phone brand fan pages on Facebook in India have been investigated. The mobile phone industry is a rapidly developing field of study for various smartphone brands adopts different marketing smartphone manufacturers’ efforts to foster positive interactions with consumers using online channels like Facebook fan sites. While the other marketing strategies have been explored earlier extensively, behaviours on Facebook fan pages is unexplored.

The data clearly demonstrate that the exchange process on social media between firms and customers is a continuous phenomenon, and organizations must ensure that customers actively participate in value creation. Marketers must recognize the cascading effect that electronic word-of-mouth may have on customers and the detrimental impact that poor eWOM can have on a specific brand. Companies must prioritize information management on social networking sites (SNSs) due to the rapid growth of online communication and its significant potential impact.

## 10. Limitation and future scope

The current study has certain drawbacks. The proposed and tested research model is an amalgamation of research models and theories relating to eWOM, trust, attitude, VCC and purchase intention. Though the proposed hypothesis was logically deductive and theoretically valid, there are some possibilities to incorporate some other constructs to the research model such as perceived usefulness (TAM), repurchase intention and product loyalty. However, based on the comprehensive review, this study has constructed limited boundaries and tested important constructs. There is a lack of research on the potential of SNSs as an instrument for the propagation of positive eWOM. This study solely examined Facebook fan pages, thus more investigation into other social media platforms (including Instagram, Twitter, Flicker, etc.) is needed to confirm the hypothesis. Only businesses with official fan pages on Facebook are included in this analysis. There is a lack of data on the total number of smartphone brand supporters on Facebook in India, this study used a non-probabilistic convenience sample technique. Due to this limitation, it is possible that the results of this study do not apply outside of this country. Geographic variation in India and elsewhere can be uncovered in future research. For the purpose of testing hypotheses, this study took a cross-sectional approach. Further studies can get more insights by conducting qualitative studies including interviews, content analysis, sentiment analysis etc.
